# The Effects of Diagnosis-Related Group Payment on Diagnostic Cerebral Angiograms through a Transradial and Transfemoral Approach: A Comparative Observational Study

**DOI:** 10.1155/2022/9670757

**Published:** 2022-01-07

**Authors:** Wei Chen, Xi-Fang Song, Min Wan, Li Liu, Wei-Hua Jia

**Affiliations:** Department of Neurology, Shijingshan Teaching Hospital of Capital Medical University, Beijing Shijingshan Hospital, Beijing 100043, China

## Abstract

**Background:**

Cerebral angiography is an X-ray examination technique widely used in hospitals. At present, it is mainly divided into two kinds of angiography examination: transfemoral artery and transradial artery puncture. The diagnosis-related group (DRG) system is a new type of payment standard recognized internationally, but its impact on medical care and health outcomes is currently controversial.

**Aim:**

In this study, we conducted a comparative study on two invasive approaches, transradial artery and transfemoral artery puncture and observed whether DRG had an impact on the quality of the medical process.

**Methods:**

We compared and analyzed patients undergoing cerebral angiography via the femoral artery and radial artery puncture by recording the relevant parameters and comfort scale scores (GCQ) during the operation, as well as postoperative complications. At the same time, we observed the proportion of different puncture routes and the success rate of cerebral angiography before and after the implementation of a DRG payment simulation.

**Results:**

The results of the comparative analysis of patients' transradial artery and transfemoral artery puncture angiography showed that the puncture success rate (99.1% vs. 97.2%, *P* > 0.05), angiography success rate (97.3% vs. 95.1%, *P* > 0.05), and X-ray radiation time (4.82 vs. 5.15 min, *P* > 0.05) demonstrated no significant difference. The ambulation time (1.52 vs. 12.06 h, *P* < 0.05), puncture time (22.42 vs. 31.02 min, *P* < 0.05), and complications (3.57% vs. 9.03%, *P* < 0.05) of the radial artery group were significantly lower than those of the femoral artery group. In contrast, the GCQ score of the radial artery group at each stage after angiography was significantly higher than that of the femoral artery group (*P* < 0.05). Compared with before the DRG simulation, the proportion of cerebral angiography with transradial artery puncture increased significantly after its implementation.

**Conclusion:**

Compared with transfemoral cerebrovascular angiography, transradial cerebrovascular angiography has many advantages, such as less local damage, less pain, less postoperative bed-rest time, significantly lower incidence of total complications, and a lower cost. Following the implementation of the DRG payment method, the quality of the angiography medical process improved.

## 1. Introduction

Diagnosis-related group (DRG) payment is based on the diagnosis of the patient's disease. Patients are divided into different groups according to their age, whether an operation is performed, whether there are comorbidities or complications, and the effect of treatment; different payment standards are then formulated for the different groups [1]. The DRG payment method has been successfully implemented in the United States, Germany, and other countries, and it is currently recognized internationally as a better payment method. The cost management control effect is unanimously recognized. However, some negative effects have also appeared in the implementation process in the above-mentioned countries, such as a reduction in expensive but necessary clinical service items, a decline in the quality of hospital services, and hindered technological progress [2]. Research on DRG payment in China started relatively late, but it has become an important measure for the country to deepen medical reform, and it represents the general trend in medical payment methods. In November 2011, Beijing took the lead in carrying out a DRG payment pilot based on basic medical insurance in six tertiary general hospitals, and the trial grouping of diseases now consists of 108 groups. Cases that meet the criteria for entry are settled according to the DRG [3].

Cerebral angiography is a new X-ray examination technology that has been widely used in clinics since the 1990s. Because it can clearly show the internal carotid artery system and vertebral basilar artery system, it has become an important examination method for patients with cerebrovascular diseases. The femoral artery extends to the external iliac artery at the midpoint of the inguinal ligament, and the puncture position through the femoral artery is 1.5∼3.0 cm below the inguinal ligament (the place with the strongest pulse) [4]. However, due to the presence of many important nerves and veins around the femoral artery, puncture and sheath placement can easily cause a series of serious complications. Therefore, this approach has certain limitations in clinical application [4]. In 1989, Campeau of Canada first reported the percutaneous puncture of the radial artery for coronary angiography. The radial artery is commonly originated from the brachial artery in the cubital fossa at the level of the neck of the radius. The pulse can be touched 2 cm from the wrist to the distal radial head. The initial puncture site of the transradial approach is at the distal end as far as possible but at least 1 cm at the proximal end of the styloid process [5]. The transradial artery puncture has the advantages of reduced complications and increased comfort, and it can also be widely used in cerebral angiography [5–7]. To this end, this study compared the safety, feasibility, and comfort of two different puncture methods in patients who underwent transradial artery puncture cerebrovascular angiography and femoral artery puncture cerebrovascular angiography, compared the proportion of different puncture routes and the success rate of cerebral angiography before and after the implementation of DRG payment simulation, and observed whether DRG payment would affect the quality of medical procedures and the application of new technologies.

## 2. Methods

### 2.1. Study Design

A total of 256 patients who underwent cerebrovascular angiography in the Department of Neurology of Beijing Shijingshan Hospital, Beijing, between January 2019 and December 2020 were selected as the research subjects. The selection criteria and groupings are shown in Figure 1. Inclusion criteria are as follows: (1) age was between 18 and 80 years; (2) after admission, there were indications of digital subtraction angiography examination by cervical vascular ultrasound, transcranial Doppler ultrasound, and head and neck computed tomography angiography examination; and (3) the patients' informed consent was obtained and approved by the hospital's medical ethics committee. Exclusion criteria are as follows: (1) history of an iodine allergy; (2) severe bleeding and/or heart, liver, kidney, and other important organ dysfunctions; (3) related examination contraindications; (4) large, unstable plaques locally; and (5) severe stenosis or occlusion of the right subclavian artery.

According to the different puncture methods, patients were divided into a radial artery group (cerebrovascular angiography via radial artery puncture, *n* = 112) and a femoral artery group (cerebrovascular angiography via femoral artery puncture, *n* = 144). There were 112 patients in the radial artery group, including 81 males (72.3%), aged 43–78 years, with an average age of 57.26 ± 3.45. There were 29 cases (25.9%) with diabetes mellitus, 72 cases (64.3%) with hypertension, and 25 cases (22.3%) with hyperlipidemia. There were 144 cases in the femoral artery group, including 107 males (74.3%), aged 47–76 years, with an average age of 59.43 ± 3.88. There were 32 cases with diabetes (28.5%), 86 cases with hypertension (59.7%), and 36 cases with hyperlipidemia (25.0%). There were no significant differences in age, sex, comorbidities, and so forth between the two groups (*P* > 0.05).

### 2.2. Variables Collected

(1) The comparison of clinical effects was mainly evaluated in relation to two factors: successful puncture, in which a radial artery sheath and femoral artery sheath were successfully inserted, and successful angiography, in which the angiography of the subclavian artery, vertebral artery, and carotid artery was successfully completed, and the branches of the supra-arch vessel and the main intracranial vessels were clearly visible [8]. (2) Comparison of the X-ray radiation time, ambulation time, and puncture time: the puncture time was measured from the beginning of disinfection and the draping of the surgical towel to the successful placement of the radial and femoral sheath. (3) Comparison of comfort: the Kolcaba comfort scale (General Comfort Questionnaire, GCQ) was used to evaluate the comfort of the two groups at 1, 6, and 12 h after the completion of the angiography. The GCQ scale score [9, 10] evaluates the four dimensions of psychology, physiology, spirituality, social culture, and environment, using the 1–4-point Likert scoring method, with a total score of 120 points. The higher the Kolcaba score, the better the patient's comfort. (4) Comparison of complication rate: the incidence of complications, such as urinary retention, hematoma, subcutaneous stasis, and venous injury and nerve injury at the puncture site were compared between the two groups. (5) The proportion of different puncture routes and the success rate of the cerebral angiography were compared before and after the implementation of the DRG payment simulation.

### 2.3. Procedure Details

1. Radial artery group: an Allen test [10] (although it is routinely not indicated anymore) was performed on the enrolled patients to check blood supply in the hands and the anastomosis between the radial artery and the ulnar artery. If the Allen test was negative, the radial artery could be punctured. The patient's right upper limb was stretched and slightly abducted, routinely disinfected, draped, and locally anesthetized with 1% lidocaine. The right radial artery was punctured using a modified Seldinger technique, and a 5F arterial sheath was inserted. The conventional catheter (A Pigtail catheter, single-bent catheter, Simon catheter, or hunter head catheter will be selected according to the needs of different patients) and guide wire were fed through the arterial sheath. The catheter tip was placed in the aortic arch, subclavian artery, vertebral artery, and carotid artery under the guidance of the guide wire, and a contrast agent was injected for the angiography. After the angiography, a compressor compressed the puncture point and removed the arterial sheath. After compressing the puncture point for 6 h, it was removed. During this period, the pressure of the compressor was released every 2 h, and the patient could get out of bed immediately after the operation (see Figure 2).
2. Femoral artery group: the patient was placed in a supine position, routinely sterilized, draped, and locally anesthetized with 1% lidocaine. The right or left femoral artery was punctured with a modified Seldinger technique, and a 5F arterial sheath was inserted. The conventional catheter and guide wire were fed through the arterial sheath, and the catheter tip was placed in the aortic arch, subclavian artery, vertebral artery, and carotid artery under the guidance of the guide wire. A contrast agent was injected for the angiography. After the operation, the arterial sheath was removed and sutured. The puncture site was pressure bandaged with an elastic bandage, and the right lower limb was immobilized for 6–8 h. The elastic bandage could be removed once the bleeding stopped (see Figure 2).

### 2.4. Statistical Analysis

SPSS 20.0 software was used for the analysis. The measurement data were expressed as mean ± standard deviation ($\overset{-}{x}$ ± *s*), and the comparison between the groups was performed with an independent sample *t*-test. The count data were expressed as a rate (%), and the comparison between the groups was performed with a chi-square test or Fisher exact probability test. *P* < 0.05 was considered statistically significant.

## 3. Results

### 3.1. Comparison of the Clinical Effects

The basic physiological data and pathological diagnosis of the patients are shown in Table 1. There was no statistical difference in age, gender, or weight between the patients in the radial artery group and the femoral artery group. In the statistical data relating to common metabolic diseases, patients with diabetes accounted for 25.9% and 28.5% in the radial artery group and the femoral artery group, respectively, and there was no statistical difference. Similarly, there was no statistical difference between the radial artery group and the femoral artery group for patients with hypertension and hyperlipidemia (hypertension: 64.3% vs. 59.7%; hyperlipidemia: 22.3% vs. 25.0%). The puncture success rate of the radial artery group was not significantly different from that of the femoral artery group (99.1% vs. 97.2%, *P* > 0.05); the angiographic success rate of the radial artery group was also not significantly different from that of the femoral artery group (97.3% vs. 95.1%, *P* > 0.05), as shown in Table 2.

### 3.2. Comparison of X-Ray Radiation Time, Ambulation Time, and Puncture Time

Compared with the femoral artery group, the radial artery group had no significant difference in X-ray radiation time (*P* > 0.05). In contrast, the ambulation time and puncture time of the radial artery group were significantly shorter than those of the femoral artery group (*P* < 0.05, Table 3 and Figure 3).

### 3.3. Changes in GCQ Score

The GCQ score of the radial artery group was significantly higher than that of the femoral artery group at 1, 6, and 12 h after angiography (*P* < 0.05, Table 4 and Figure 4).

### 3.4. Comparison of Complication Rate

The total complication rate of the radial artery group was significantly lower than that of the femoral artery group (*P* < 0.05, Table 5).

### 3.5. Compared with before the DRG Payment Simulation

The proportion of cerebral angiography in the transradial artery group increased significantly after its implementation (*P* < 0.05, Table 6), and the success rate of the angiography did not change significantly (*P* > 0.05, Table 6).

## 4. Discussion

Cerebral angiography is a minimally invasive X-ray examination technique widely used in neurology departments. It has become the gold standard for the diagnosis of cerebrovascular diseases due to its accuracy, intuition, dynamics, and mature technology. However, different puncture approaches not only affect the impact of angiography but also have different levels of safety. The transfemoral approach was performed at 1.5∼3.0 cm below the inguinal ligament using the modified Seldinger technique, which has always been the classic method for cerebral angiography. However, it is not easy to stop bleeding, and there are many puncture-related complications [11–13]. Therefore, in recent years, as a new technique, transradial artery puncture cerebral angiography has gradually been applied in clinical practice. The initial puncture site of the transradial approach is at the distal end as far as possible but at least 1 cm at the proximal end of the styloid process. For example, Matsumoto performed cerebral angiography via the radial approach with a 4F catheter, in which 98% of patients were successful using a superselective internal carotid artery and 95% of patients were successful using a superselective vertebral artery [14].

From the analysis of clinical effects, first, this study found that the radial artery group demonstrated no significant difference in the success rate of the puncture, the success rate of the angiography, and the X-ray radiation time compared with the femoral artery group. In a study on the amount of X-ray radiation exposure received by a surgeon during an operation, Son et al. [15] found that the fluoroscopy time of the radial artery group and the femoral artery group was 9.4 and 10.3 min (*P*=0.70), and the difference was not statistically significant. The results of these two studies are also consistent with our results, inicatidng that the success rate of angiography in the radial artery group and the femoral artery group is similar without increasing the amount of X-ray radiation exposure received by the surgeon. Second, the ambulation time of the radial artery puncture group was significantly shorter than that of the femoral artery group. As we know, staying in bed for a long time can easily cause the blood in the patient's lower limbs to enter into a state of hypercoagulability, especially in elderly patients, and it easily forms deep vein thrombosis. However, the shorter the time of immobilization in bed after an operation, the earlier a patient can move around, which has a positive significance in reducing the occurrence of complications such as deep vein thrombosis of the lower limbs. At the same time, patients in the transradial artery group only need to wear a compression device for about 6 h, which is convenient for nursing care. In the femoral artery group, the puncture site needs to be pressurized with an elastic bandage, and the puncture side of the lower limb is immobilized for 6–8 h. After the operation, it is necessary to observe whether the dorsal artery is pulsating, and the amount of nursing care required by the patient is greatly increased. Third, the puncture time of the radial artery group was significantly shorter than that of the femoral artery group, and the GCQ score was significantly higher after the completion of the angiography, indicating that the radial artery group was more comfortable. The reduction in puncture time can effectively reduce operation time, improving the patient's tolerance and their compliance. As for the radial artery approach, there is no need for skin preparation at the perineum, thereby reducing the patient's psychological discomfort. It is therefore easier for patients to agree to the examination, which is of great help in improving the clinical diagnosis, evaluation, and treatment of cerebrovascular diseases. Fourth, compared with the femoral artery group, the total complication rate of the radial artery group was significantly lower than that of the femoral artery group. Moreover, even if the patients undergoing interventional surgery through the radial artery had surgical complications, the majority had a radial artery spasm and bleeding at the puncture port, with mild symptoms that were easy to handle. However, other adverse reactions and common operative complications were significantly less than in patients with the femoral artery approach. In particular, the incidence of venous and nerve injury at the puncture site was significantly lower than that in the femoral artery group, which is closely related to the anatomical characteristics of the radial artery and femoral artery [11]. The radial artery is relatively shallow and can be easily compressed to stop bleeding, while the femoral artery is relatively deep. It is relatively difficult to stop bleeding by pressing the puncture site after the operation, which is more likely to damage the femoral vein and femoral nerve, leading to local massive hemorrhage, subcutaneous hematoma, and other complications [16]. Furthermore, because of the longer time spent in bed in the transfemoral artery group, the incidence of urinary retention was also higher than in the transradial artery group. Fifth, compared to before the DRG payment simulation, the proportion of cerebral angiography procedures in the radial artery group increased significantly after its implementation, and the success rate of the angiography did not change significantly. We know that DRG payment is to divide patients into different groups and formulate different payment standards for different groups [1], which has a significant impact on improving medical efficiency, reducing hospitalization costs, and shortening the length of stay. Although there are no comparative statistics on the length of stay and cost of the two approaches for cerebral angiography, there have been many statistical studies on the comparison of these two different approaches in terms of coronary intervention treatment [17–19]. The hospitalization time and cost for patients undergoing interventional therapy via the radial artery approach are less than for patients who choose the femoral artery approach [17, 20]. Studies have shown that after the implementation of DRG payment, the average cost, examination, laboratory, and hospitalization costs were reduced [21]. Therefore, in the case of no significant difference in surgical effect, patients are more willing to choose the transradial approach with less hospital stay and lower cost, which indirectly improve the diagnostic efficiency of cerebrovascular diseases. This is also confirmed by our research. After the DRG payment trial, the proportion of cerebral angiography procedures in the transradial artery group increased significantly. This demonstrates that DRG payment has a positive effect on improving the quality of the medical process of cerebral angiography and the application of the new technology for transradial cerebral angiography.

However, this study only focused on the effect of a DRG payment simulation at a medical institution in Beijing, and the time span of the data needs to be expanded. A simulated operation does not completely represent a real-life DRG operation, and long-term follow-up research is needed to explore the actual operation effect of DRG payment.

## 5. Conclusion

In summary, we can see that compared with transfemoral cerebrovascular angiography, the success rate of transradial cerebrovascular angiography is similar, and the amount of X-ray radiation exposure received by the surgeon is not increased. In addition, patients have less local injury, spend less time in bed after surgery, and can take care of themselves in their daily lives, which makes them feel better, and significantly improves their tolerance. The overall complication rate is significantly reduced, the length of hospital stay is shortened, and the cost is reduced. Following the DRG payment trial, the proportion of procedures using the new technique for transradial cerebrovascular angiography increased significantly, thus demonstrating that DRG payment has a positive effect on improving the quality of the cerebral angiography medical process and the application of the new transradial cerebral angiography technology. The advantages described above indicate that transradial cerebrovascular angiography meets the conditions for the promotion of the new diagnosis and treatment technology in clinical practice.

## Figures and Tables

**Figure 1:** Flowchart depicting the comparative analyses performed. DCA: diagnostic cerebral angiogram.

**Figure 2:** Procedure details.

**Figure 3:** Bar graph showing the radiation exposure time, time for getting out of bed after surgery (h), and procedure duration. Data are shown as mean ± SD,  ^*∗*^*P* < 0.05.

**Figure 4:** Bar graph showing the GCQ score at different times after surgery. Data are shown as mean ± SD,  ^*∗*^*P* < 0.05.

**Table 1:** Baseline characteristics and outcomes for patients: transradial versus transfemoral approach for cerebral angiograms.

Variables	Transradial approach	Transfemoral approach	*P* value
Patients, *n*	112	144	
Age, mean ± SD, years	57.2 6 ± 3.45	59.43 ± 3.88	0.21
Gender (%)			0.72
Male	81 (72.3)	107 (74.3)	
Female	31 (27.7)	37 (25.7)	
Weight, kg, mean ± SD	72.6 ± 8.7	69.3 ± 10.2	0.44
Diabetes mellitus, *n* (%)	29 (25.9)	32(28.5)	0.48
Hypertension, *n* (%)	72 (64.3)	86 (59.7)	0.46
Hyperlipidemia, *n* (%)	25 (22.3)	36 (25.0)	0.62

**Table 2:** Comparison of clinical effects of the two groups.

Group	Number of cases	Puncture success	Angiographic success
Radial artery group	112	111 (99.1%)	109 (97.3%)
One attempt	78	78 (69.6%)	77 (68.8%)
Two attempts	34	33 (29.5%)	32 (28.5%)
Femoral artery group	144	140 (97.2%)	137 (95.1%)
One attempt	93	93 (64.6%)	92 (63.9%)
Two attempts	51	47 (32.6%)	45 (31.2%)
*P* value		0.28	0.37

**Table 3:** Comparison of X-ray radiation time, hospital stay, and puncture time of the two groups ($\bar{x}\pm s$).

Group	X-ray radiation time (min)	Ambulation time (h)	Puncture time (min)
Radial artery group (*n* = 112)	4.82 ± 1.13	1.52 ± 0.86	22.42 ± 3.55
Femoral artery group (*n* = 144)	5.15 ± 1.01	12.06 ± 4.23	31.02 ± 2.71
*P* value	0.76	<0.001	<0.001

**Table 4:** Changes in GCQ score of the two groups ($\bar{x}\pm s$).

Group	1 h score after angiography	6 h score after angiography	12 h score after angiography
Radial artery group (*n* = 112)	50.15 ± 6.32	77.84 ± 8.29	91.03 ± 5.88
Femoral artery group (*n* = 144)	42.56 ± 7.23	60.63 ± 6.28	75.47 ± 6.72
*P* value	<0.001	<0.001	<0.001

**Table 5:** Comparison of complication rate (*P*=0.038).

Group	Urinary retention	Hematoma	Subcutaneous stasis	Vasospasm	Vein injury at the puncture site	Nerve injury at the puncture site	Total complication rate
Radial artery group (*n* = 112)	0	0	3	1	0	0	4 (3.57%)

Femoral artery group (*n* = 144)	3	2	5	0	1	2	13 (9.03%)

**Table 6:** Proportion of puncture routes and success rate of angiography before and after the implementation of DRGs payment simulation.

Group	Number of cases	Radial artery puncture	Radiography success
Before the implementation of DRGs payment simulation	152	50 (32.9%)	145 (95.4%)
After the implementation of DRGs payment simulation	104	62 (59.6%)	101 (97.1%)
*P* value		<0.001	0.49

## Data Availability

The datasets used and analyzed during the current study are available from the corresponding author on reasonable request.
